# Pretreatment with Shenmai Injection Protects against Coronary Microvascular Dysfunction

**DOI:** 10.1155/2022/8630480

**Published:** 2022-06-09

**Authors:** Zhaohai Zheng, Zhangjie Yu, Buyun Xu, Yan Zhou, Yangbo Xing, Qingsong Li, Weiliang Tang, Fang Peng

**Affiliations:** ^1^Department of Cardiology, Shaoxing People's Hospital (Shaoxing Hospital, Zhejiang University School of Medicine), Shaoxing 312000, Zhejiang, China; ^2^Zhejiang University School of Medicine, Hangzhou 310000, Zhejiang, China; ^3^Shaoxing University School of Medicine, Shaoxing 312000, Zhejiang, China; ^4^Department of Cardiology, Awati County People's Hospital, No.1 North Jiefang Road, Awati County, Xinjiang Uygur Autonomous Region 843000, China

## Abstract

**Background:**

The clinical treatment of coronary microvascular dysfunction (CMD) is mainly based on conventional medicine, but the mechanism of the medicine is single and the efficacy is different. Shenmai injection (SMI) has a variety of ingredients, but the effect of SMI on CMD has not been studied. This study investigated the effect of SMI on CMD and its possible mechanism.

**Methods:**

The protective effect of SMI on CMD was evaluated in Sprague-Dawley (SD) rats and human umbilical vein endothelial cells (HUVECs). In vivo, forty-five male SD rats were randomly divided into control group (sham group), CMD group (model group), and SMI group (treatment group). Two weeks after SMI intervention, laurate was injected into the left ventricle of rats to construct a CMD model. Blood samples were collected to detect myocardial enzymes, oxidative stress, and inflammatory factors, and the hearts of rats were extracted for histopathological staining and western blot detection. In vitro, a hydrogen peroxide-induced endothelial injury model was established in HUVECs. After pretreatment with SMI, cell viability, oxidative stress, vasodilative factors, and apoptosis were detected.

**Results:**

In vivo, pretreatment with SMI could effectively reduce the concentrations of lactate dehydrogenase (LDH), creatine kinase-MB (CK-MB), cardiac troponin I (cTnI), endothelin-1 (ET-1), tumor necrosis factor alpha (TNF-*α*), interleukin 6 (IL-6), and malondialdehyde (MDA) in the serum of rats. Meanwhile, the expression of bcl-2-associated X (Bax) and caspase-3 protein in the myocardium of rats was decreased in the SMI group. The levels of nitric oxide (NO) and superoxide dismutase (SOD) and the expression of B-cell lymphoma-2 (Bcl-2) were higher in the SMI group than in the CMD group. Pathological staining results showed that SMI could effectively reduce inflammatory infiltration and the formation of collagen fibers and microthrombus in the rat myocardium. In vitro, intervention with SMI could improve endothelial function in a dose-dependent manner as evidenced by increasing the activity of endothelial cells and the expression of NO, SOD, endothelial nitric oxide synthase (eNOS), and Bcl-2, while decreasing cell apoptosis and the levels of ET-1, MDA, Bax, and caspase-3.

**Conclusions:**

Pretreatment with SMI could improve CMD by alleviating oxidative stress, inflammatory response, and apoptosis and then improving vascular endothelial function and microvascular structure.

## 1. Introduction

Coronary atherosclerotic heart disease is an important disease leading to myocardial ischemia. Its typical pathological changes are epicardial coronary atherosclerosis and vascular stenosis. However, studies have shown that about 66% of women and 33% of men with chest pain and a few patients with acute myocardial infarction show no significant structural coronary disease on angiography [1]. These patients may be affected by coronary microvascular dysfunction (CMD). In the coronary circulation, arterioles and anterior arterioles with a diameter of less than 500 *μ*m constitute the coronary microcirculation, and CMD is usually defined as increased resistance and/or impaired vascular dilation of the microvasculature, resulting in myocardial hypoperfusion during stress [2, 3]. CMD is closely associated with ischemic cardiomyopathy, acute coronary syndrome, sudden cardiac death, and other serious adverse events [4, 5].

At present, CMD is considered to be a complex pathophysiological process mediated by multiple factors and multiple steps, and the main mechanism is the abnormal structure or function of the coronary microvasculature. An abnormal microvascular structure is mainly manifested as lumen obstruction, vascular remodeling, decreased vascular area, and perivascular fibrosis [6, 7]. Microvascular dysfunction can be divided into endothelium-dependent and nonendothelium-dependent, among which the endothelium-dependent dysfunction is the main one.

At the moment, the clinical treatments of CMD mainly include nicorandil, statins, nitric acid esters, and angiotensin-converting enzyme inhibitors, and other drugs. Nevertheless, these drugs can only improve the myocardial blood supply through a single mechanism, and the efficacy of CMD is somewhat deficient. Shenmai injection (SMI) is a kind of traditional Chinese medicine with various ingredients, mainly composed of Radix Ginseng Rubra and Radix Ophiopogon [8, 9]. Ophiopogonin D is one of the main active components of Radix Ginseng, which can rescue apoptosis by alleviating mitochondrial damage of myocardial cells [10]. Moreover, previous studies have shown that SMI can improve cardiac microcirculation by eliminating oxygen free radicals [11]. At the same time, SMI can also protect the myocardium or cardiomyocytes of rats from ischemia-reperfusion injury by stabilizing intracellular Ca^2+^ homeostasis, maintaining mitochondrial homeostasis and improving energy metabolism [12–15]. However, the therapeutic effect of SMI on CMD has not been reported. The purpose of our study was to investigate the effect of SMI on CMD improvement and its possible protective mechanism.

## 2. Materials and Methods

### 2.1. Drugs and Reagents

SMI was purchased from Zhengda Qing Chun Bao Pharmaceutical Co. Ltd. (Hangzhou, China). All cell culture products were purchased from Gibco (Grand Island, NY, USA). Sodium laurate and sodium carboxymethyl cellulose were purchased from MedChemExpress LLC (Shanghai, China). Hydrogen peroxide (H_2_O_2_) was purchased from Shandong Lierkang Medical Technology Co. Ltd. (Shandong, China). Bcl-2 antibody, Bax monoclonal antibody, caspase-3 antibody, endothelial nitric oxide synthase (eNOS) polyclonal antibody, and glyceraldehyde-3-phosphate dehydrogenase (GAPDH) monoclonal antibody were all purchased from Proteintech (Proteintech Group, Wuhan, China).

### 2.2. Animals and Treatment

Forty-five male Sprague-Dawley (SD) rats weighing 300–350 g (purchased from Laboratory Animal Research Center of Zhejiang Chinese Medical University, Hangzhou, China) were kept in cages and provided with free water and food. We kept these rats in a standard environment with a humidity of 55 ± 5% and temperature of 22 ± 2°C.

Rats were randomly divided into three groups: control group (sham group), CMD group (model group), and SMI group (treatment group), with 15 rats in each group. Rats in the drug intervention group were intramuscular injected with SMI (0.24 ml/kg, i.m.) for 2 weeks. Rats in CMD and control groups were administered with saline (0.24 ml/kg, i.m.). 12 h after the final treatment, we used pentobarbital sodium (40 mg/kg, i.p.) to anesthetized rats. Rats were fixed in supine position, and the heart and aortic arch were exposed by opening the chest at the second and third ribs. During 30 s of blocking the ascending aorta, the left ventricle of rats in CMD and SMI groups was injected with sodium laurate (2 g/L, 0.2 mL) to construct a microvascular injury model [16, 17], and the control group received an equal volume of saline to simulate the experimental process. All rats were sacrificed 24 h after thorax closure. Blood from the abdominal aorta of rats was extracted for subsequent analysis. The hearts of each group were extracted for subsequent histopathological and western blot analysis.

### 2.3. Measurement of Myocardial Enzyme Profile

The serum levels of lactate dehydrogenase (LDH), creatine kinase-MB (CK-MB), and cardiac troponin I (cTnI) were determined using an automatic biochemical analyzer (Abbott Aeroset TM, USA).

### 2.4. Detection of Vascular Endothelial Function

The nitric oxide (NO) assay kit (Beyotime Biotechnology, Shanghai, China) and endothelin-1 (ET-1) enzyme-linked immunosorbent assay (ELISA) kit (Cloud-Clone Technology, Wuhan, China) were used to detect the content of NO and ET-1 under the instructions of the manufacturer.

### 2.5. Detection of Oxidative Stress Levels and Inflammation Cytokines

The levels of malondialdehyde (MDA) and superoxide dismutase (SOD) were measured by using the respective assay kits (Beyotime Biotechnology, Shanghai, China). The serum levels of interleukin 6 (IL-6) and tumor necrosis factor alpha (TNF-*α*) were detected using ELISA assay kits (Cloud-Clone Technology, Wuhan, China).

### 2.6. Myocardial Pathological Staining

The heart tissue was fixed, dehydrated and embedded, and then cut into 5 *μ*m slices. Histopathological analysis was performed with hematoxylin-eosin (HE) staining (Senbeijia Biotechnology, Nanjing, China), Masson's trichrome staining (Senbeijia Biotechnology), and Carstairs staining (GenMed Scientific Inc, USA).

### 2.7. Cell Culture and Treatment

Human umbilical vein endothelial cells (HUVECs) were purchased from iCell (iCell Bioscience Inc, Shang, China). Briefly, HUVECs were cultured in endothelial cell medium (ECM; Sciencell Research Laboratories, CA, USA) with the addition of 5% fetal bovine serum, 1% penicillin/streptomycin, and 1% endothelial cell growth supplement. The cells were maintained at 37°C in a humidified incubator containing 5% CO_2_. SMI was diluted to different concentrations with ECM. H_2_O_2_ was diluted to 0.6 mM with ECM.

In order to explore the toxic effect of SMI on HUVECs, we pretreated HUVECs with SMI (0, 0.5%, 1%, 5%, 10%, 20%, 30%, 50%) for 12 h. Results of cell viability showed that the concentration of SMI should be less than 20%. Then, for selecting the most suitable concentration of intervention of SMI, we pretreated HUVECs with SMI (0, 1%, 2%, 2.5%, 3%, 4%, 5%) for 12 h and then treated with H_2_O_2_ (0.6 mM) for 2 h to induce an endothelial cell injury model [18, 19]. According to the test of cell viability, we decided to incubate HUVECs with SMI at the concentrations of 1% and 5% in the further study. Then, HUVECs were pretreated with SMI (1%, 5%) for 12 h and H_2_O_2_ for 2 h as mentioned above, and the medium and cells were collected for the following test.

### 2.8. Cell Viability

Cell viability was examined by cell counting kit-8 (CCK8) assay (Beyotime Biotechnology, Shanghai, China). After being cultured with H_2_O_2_, HUVECs were incubated with CCK8 solution (10 *μ*L/100 *μ*L medium) for 2 h. The absorbance was measured at 450 nm with an automatic microplate reader (SpectraMax Plus, USA).

### 2.9. Detection of Vasodilative Factors and Oxidative Stress of HUVECs

The concentrations of NO and ET-1 in the cell supernatant were detected using an NO assay kit (Beyotime Biotechnology, Shanghai, China) and Human ET-1 ELISA kit (Cloud-Clone Technology, Wuhan, China), respectively. The detection method of SOD and MDA content in the cells was shown as above.

### 2.10. Terminal Deoxynucleotidyl Transferase Mediated dUTP Nick End Labeling (TUNEL) Staining

Apoptosis was detected by using TUNEL assay (Beyotime Biotechnology, Shanghai, China). The nuclei were stained again with 4,6-diamino-2-phenylindole (DAPI; Beyotime Biotechnology, Shanghai, China). Three random regions of each group of cells were observed under a fluorescence microscope (Leica, DE).

### 2.11. Western Blotting (WB)

The total protein of rat myocardium or HUVECs was extracted with cold lysate containing protease inhibitors and centrifuged at 4°C at 12000 × *g* for 5 min. The concentration of extracted protein was detected by the BCA method, and the protein was fully mixed with 5x loading buffer and then boiled at 100°C for 5 min for denaturation. Equal amounts of protein (30 *μ*g) from rats and HUVECs were separated via sodium dodecyl sulfate-polyacrylamide gel electrophoresis and transferred to polyvinylidene fluoride membranes (Merck Millipore Ltd, IRL, UK) using a transblot apparatus. The membranes were blocked in sealing fluid for 2 h and then placed on a shaker and incubated at 4°C overnight with specific primary antibodies against Bax (1 : 1000), caspase-3 (1 : 1000), Bcl-2 (1 : 1000), eNOS (1 : 1000), and GAPDH (1 : 1000). The membranes were then incubated with anti-rabbit and anti-rat secondary antibodies (1 : 2000) for 2 h. After cleaning the strip with TBST solution, a luminescent solution was added and then it was put under an ECL system for observation.

### 2.12. Statistical Analysis

All values were expressed as means ± standard deviation (SD). One-way analysis of variance followed by least significant difference method was applied to analyzing the differences among groups. Statistical significance was accepted as *P* < 0.05.

## 3. Result

### 3.1. SMI Improves Laurate-Induced CMD in Rats

Sodium laurate was injected into the left ventricle of the rats to mimic CMD. SMI was utilized as pretreatment. As shown in Figures 1(a)–1(c), the concentrations of LDH, CK-MB, and cTnI were significantly rising in the CMD group (*P* < 0.01). Compared with the CMD group, there was a dramatic decline in the levels of LDH, CK-MB, and cTnI in the SMI group (*P* < 0.01, *P* < 0.05).

Rats in the CMD group had a clearly increased level of TNF-*α* and IL-6 in serum compared with those in the control group (*P* < 0.01). In contrast with the CMD group, the SMI group exhibited a significant decrease in the level of TNF-*α* and IL-6 in serum (*P* < 0.01) (Figures 2(a) and 2(b)).

Histopathological examination was performed by HE, Masson's trichrome, and Carstairs staining to intuitively detect myocardial injury. The results of HE staining implied that myocardial cells in the CMD group were damaged and disordered, accompanied by inflammatory cell infiltration, while those changes were significantly improved in the SMI group (Figure 3). As can be seen from the results of Masson's trichrome staining, laurate could cause the hyperplasia of collagen fibers between myocardial fibers, and SMI could effectively alleviate this process (Figure 4). In Carstairs staining, microthrombus was observed in the microvasculature of rats in the CMD group, but rats in the SMI group had less microthrombus formation in their microvasculature (Figure 5).

### 3.2. SMI Inhibits Apoptosis of Rat Cardiomyocytes and HUVECs

In HUVECs, the results of CCK8 tests showed that a low SMI concentration (1%–20%) would not change the cell viability of HUVECs, while when SMI concentration was greater than 20%, the cell viability of HUVECs decreased significantly (*P* < 0.01, Figure 6(a)). Therefore, the SMI concentration of cells cultured in subsequent tests should be less than 10%.

So as to further explore the function of SMI concentration on cell injury and apoptosis, we had intervened HUVECs with different concentrations of SMI. The results of cell viability test showed that H_2_O_2_ could significantly reduce cell viability, and SMI could improve this injury to a certain extent in a dose-dependent manner (*P* < 0.01, *P* < 0.05, Figure 6(b)).

In line with the above results, TUNEL staining showed that H_2_O_2_ could induce nuclear pyknosis and apoptosis of HUVECs, while SMI could alleviate nuclear changes and apoptosis (Figure 6(c)).

The antiapoptotic effect of SMI was more obvious in results of WB. As shown in Figure 6(d), H_2_O_2_ could increase the expression of Bax, caspase-3, and other apoptotic proteins, while decreasing the expression of Bcl-2. SMI could effectively reverse this process (*P* < 0.01). Interestingly, H_2_O_2_ would decrease the expression of eNOS, while intervention of SMI could increase the expression of eNOS (*P* < 0.01).

The results of WB in rats' myocardium also showed that SMI could inhibit apoptosis and promote the antiapoptosis process, mainly by decreasing the expression of Bax and caspase-3 and increasing the expression of Bcl-2 (*P* < 0.01, Figure 6(e)).

### 3.3. SMI Suppresses Superoxide Formation in CMD Rats and HUVECs

The levels of oxidative stress in rats in the CMD group were measured by MDA and SOD. CMC-Na caused a marked elevation in the level of MDA and a distinct reduction in SOD (*P* < 0.01, Figure 7(a)). The level of MDA was reduced and the level of SOD was elevated when rats were treated with SMI (*P* < 0.01, Figure 7(b)).

In HUVECs, H_2_O_2_ caused an obvious decline in SOD and a significant growth in MDA (*P* < 0.01). SMI alleviated this phenomenon in a dose-dependent manner (*P* < 0.01, Figures 7(c) and 7(d)).

### 3.4. SMI Improves Endothelial Cell Function in CMD Rats and HUVECs

As shown in Figures 8(a) and 8(b), the level of NO in rats in the CMD group was decreased, while the level of ET-1 was increased compared with the control group (*P* < 0.01, *P* < 0.05). SMI could increase the synthesis of NO and decrease the production of ET-1 in rats with CMD.

Similar to the above, when endothelial injury happened, the production of NO of endothelial cells decreased and the synthesis of ET-1 increased. Intervention of SMI could effectively improve endothelial function by promoting the synthesis of NO and inhibit the production of ET-1 in endothelial cells (*P* < 0.01, Figures 8(c) and 8(d)).

## 4. Discussion

CMD is a clinical syndrome of myocardial ischemia caused by structural and/or functional abnormalities of coronary microvasculature (anterior arterioles and arterioles, diameter <500 *μ*m) under the influence of various pathogenic factors. In 2013, the Task Force on the management of stable coronary artery disease of the European Society of Cardiology officially named the disease as coronary microvascular dysfunction [20]. The pathogenesis of CMD is a complex pathological and physiological process. Modern pharmacological studies have found that SMI can increase myocardial blood perfusion and improve myocardial hypoxia through multiple pathways and mechanisms with various components [21, 22]. Both in vivo and in vitro, our research demonstrated the protective effect of SMI on CMD. Our results further suggested that the protective mechanisms might be the improvement of endothelial dysfunction, reduction of myocardial inflammatory response, and reduction of oxidative stress and apoptosis.

In this study, the CMD model of rats was established by injecting laurate into the left ventricle of rats. The results of pathological staining showed that the myocardial cells in the model group were disordered, inflammatory cells were infiltrated, and microthrombus was formed, manifesting that the CMD model was successfully constructed. Compared with the CMD group, the infiltration of inflammatory cells and collagenous fibers in myocardial fibers was decreased, and the formation of microthrombus in coronary microvasculature was decreased in the SMI group. These results suggested that SMI could ameliorate the disorder of cell arrangement, help improve the cooperative contraction of myocardium, and then improve the cardiac function. At the same time, SMI alleviated the formation of coronary microvascular microthrombus and contributed to improving the blood supply of myocardial microcirculation. Meanwhile, in the SMI group, the levels of LDH, CK-MB, and cTnI, which reflecting myocardial ischemia or myocardial infarction, were also significantly reduced [23]. These results suggested that preconditioning with SMI could effectively improve the changes of coronary microvascular structure and effectively prevent myocardial injury caused by myocardial ischemia.

In addition to the reconstruction of coronary microvascular structure, CMD was mainly associated with microvascular dysfunction. Microvascular dysfunction is characterized by impaired microvascular systolic/diastolic function, which can be classified into endothelial cell-dependent and nonendothelial cell-dependent dysfunction [24]. Endothelial cell-dependent dysfunction is often characterized by reduced synthesis and increased degradation of NO. NO, synthesized by substrate L-arginine in the presence of eNOS, mediates vasodilation by promoting calcium sensitivity and adenosine triphosphate (ATP)-dependent potassium channel opening [2]. Nonendothelium-dependent dysfunction is generally manifested as metabolic disorders of ET-1, which induces the contraction of vascular smooth muscle and leads to excessive contraction of microvasculature by being combined with the corresponding receptor on vascular smooth muscle [25]. Similar to these conclusions, our results suggested that SMI could promote the synthesis of NO and reduce the generation of ET-1 so as to effectively improve the microvascular dysfunction. And the mechanism might be related to the increase of eNOS expression.

CMD is always related to elevated oxidative stress and decreased antioxidant capacity [26]. When the oxidative stress is overactivated, superoxide anion reacts with NO to form nitrite, leading to the degradation of NO [27, 28] and inducing endothelial cell migration, angiogenesis dysfunction, and abnormal repair vascular proliferation [29]. It was proved in our research that SMI could reduce MDA and increase SOD to control the level of oxidative stress of the system both in vivo and in vitro.

Inflammatory response is a relatively new risk factor for cardiovascular disease and is attracting more and more attention. Studies have shown that IL-6, white blood cells, and highly sensitive C-reactive protein (hs-CRP) in the peripheral blood of patients with CMD were significantly higher than those of healthy patients [30]. Other experiments have proved that high levels of CRP were negatively correlated with myocardial perfusion [31]. This was consistent with our observation that the levels of IL-6, TNF-*α*, and other inflammatory factors were increased in rats with CMD, which were attenuated by SMI to some extent. The potential mechanism might be that inflammatory factors could damage the vascular endothelium, activate endothelial cells to release endothelin and endothelin-like immune complexes, reduce the release of NO and prostacyclin, and lead to abnormal endothelial diastolic function. At the same time, inflammation activated the oxidative stress of the system, stimulated the abnormal proliferation of endothelial cells, thickened the intima, and affected the structure and function of the endothelium [31].

Oxidative stress and inflammation will lead to apoptosis of vascular endothelial cells, and apoptosis in turn affects the former. The study of Wang et al. [32] showed that when CMD occurred, the expression of apoptotic protein such as caspase-3 and Bax increased, while the level of antiapoptotic factor Bcl-2 decreased. TUNEL staining showed that SMI could effectively relieve apoptosis. The results of WB showed that pretreatment with SMI could decrease the expression of apoptotic factors like Bax and caspase-3 and increase the expression of Bcl-2.

Firstly, this study confirmed that SMI could improve CMD in a variety of ways; however, only animal and cell experiments were observed, and no clinical effects were observed. Secondly, the specific cellular pathways which SMI improves CMD have not been thoroughly studied. In addition, the sample size of cells studied is too small. Therefore, further research will be needed to address these limitations.

## 5. Conclusion

Overall, this article demonstrated that pretreatment with SMI could improve CMD both in vivo and in vitro. We hypothesized that the mechanism might be related to reducing oxidative stress, inflammatory response, and apoptosis and then promoting the release of NO, improving endothelial cell function, and improving vascular structure abnormalities.

## Figures and Tables

**Figure 1:** Effects of SMI on serum LDH (a), CK-MB (b), and cTnI (c) levels in CMD rats. Data are expressed as mean ± SD (*n* = 5). ^*∗∗*^*p* < 0.01 vs. control group; ^#^*p* < 0.05, ^##^*p* < 0.01 vs. CMD group.

**Figure 2:** Effects of SMI on serum inflammatory indexes TNF-*α* (a) and IL-6 (b) in CMD rats. Data are expressed as mean ± SD (*n* = 5). ^*∗∗*^*p* < 0.01 vs. control group; ^##^*p* < 0.01 vs. CMD group.

**Figure 3:** HE pathological staining of myocardial tissue in CMD rats. (a) Control group. (b) CMD group. (c) SMI group. The black arrows represent inflammatory fine infiltrates (×200; scale bar = 100 *μ*m).

**Figure 4:** Masson's trichrome staining of myocardial tissue in CMD rats. (a) Control group. (b) CMD group. (c) SMI group. The black arrows represent the extracellular fibroplasia of myocardium. (×200; scale bar = 100 *μ*m).

**Figure 5:** Carstairs staining of myocardial tissue in CMD rats. (a) Control group. (b) CMD group. (c) SMI group. The black arrows represent the formation of microthrombus between myocardial cells (×200; scale bar = 100 *μ*m).

**Figure 6:** Effects of SMI on cell viability and apoptosis. (a) The effect of SMI on HUVECs viability. (b) Effects of different concentrations of SMI on the decreased cell viability induced by H_2_O_2_. (c) TUNEL staining of HUVECs. The white arrows represent apoptotic nuclei (×100; scale bar = 100 *μ*m). (d) Western blot analysis of Bax, caspase-3, Bcl-2, and eNOS in HUVECs. (e) Western blot analysis of Bax, caspase-3, Bcl-2 in rats' myocardium. Data are expressed as mean ± SD (*n* = 5). ^*∗∗*^*p* < 0.01 vs. control group; ^#^*p* < 0.05, ^##^*p* < 0.01 vs. CMD group.

**Figure 7:** Effects of SMI on MDA (a) and SOD (b) in serum of CMD rats. Effects of SMI on MDA (c) and SOD (d) in HUVECs. Data are expressed as mean ± SD (*n* = 5). ^*∗∗*^*p* < 0.01 vs. control group; ^##^*p* < 0.01 vs. CMD group.

**Figure 8:** Effects of SMI on serum NO (a) and ET-1 (b) in CMD rats. Effects of SMI on NO (c) and ET-1 (d) in the supernatant of HUVECs. Data are expressed as mean ± SD (*n* = 5). ^*∗∗*^*p* < 0.01 vs. control group; ^#^*p* < 0.05, ^##^*p* < 0.01 vs. CMD group.

## Data Availability

All data sets presented in this study are available from the corresponding authors on reasonable request.

## Abbreviations

CMD: Coronary microvascular dysfunction
SMI: Shenmai injection
H_2_O_2_: Hydrogen peroxide
Bcl-2: B-cell lymphoma-2
Bax: Bcl-2-associated X
eNOS: Endothelial nitric oxide synthase
GAPDH: Glyceraldehyde-3-phosphate dehydrogenase
SD: Sprague-Dawley
LDH: Lactate dehydrogenase
CK-MB: Creatine kinase-MB
cTnI: Cardiac troponin I
NO: Nitric oxide
ET-1: Endothelin-1
MDA: Malondialdehyde
SOD: Superoxide dismutase
IL-6: Interleukin 6
TNF-*α*: Tumor necrosis factor alpha
HE: Hematoxylin-eosin
HUVECs: Human umbilical vein endothelial cells
ECM: Endothelial cell medium
CCK8: Cell counting kit-8
TUNEL: Terminal deoxynucleotidyl transferase mediated dUTP nick end labeling
WB: Western blot
SD: Standard deviation
hs-CRP: Highly sensitive C-reactive protein.
